# Upbeat: Augmented Reality-Guided Dancing for Prosthetic Rehabilitation of Upper Limb Amputees

**DOI:** 10.1155/2019/2163705

**Published:** 2019-03-19

**Authors:** Marina Melero, Annie Hou, Emily Cheng, Amogh Tayade, Sing Chun Lee, Mathias Unberath, Nassir Navab

**Affiliations:** ^1^Medical Physics and Biomedical Engineering, University College London, London WC1E 6BT, UK; ^2^Department of Computer Science, Johns Hopkins University, Baltimore 21218-2683, USA

## Abstract

Unsuccessful rehabilitation therapy is a widespread issue amongst modern day amputees. Of the estimated 10 million amputees worldwide, 3 million of whom are upper limb amputees, a large majority are discontent and experience rejection with their current prosthesis during activities of daily living (ADL). Here we introduce *Upbeat*, an augmented reality (AR) dance game designed to improve rehabilitation therapies in upper limb amputees. In *Upbeat*, the patient is instructed to follow a virtual dance instructor, performing choreographed dance movements containing hand gestures involved in upper limb rehabilitation therapy. The patient's position is then tracked using a Microsoft Kinect sensor while the hand gestures are analyzed using EMG data collected from a Myo Armband. Additionally, a gamified score is calculated based on how many gestures and movements were correctly performed. Upon completion of the game, a diagnostic summary of the results is shown in the form of a graph summarizing the collected EMG data, as well as with a video displaying an augmented visualization of the patient's upper arm muscle activity during gameplay. By gamifying the rehabilitation process, *Upbeat* has the potential to improve therapy on upper limb amputees by enabling the start of rehabilitation immediately after trauma, providing personalized feedback which professionals can utilize to accurately assess patient's progress, and increasing patient excitement, therefore increasing patient willingness to complete rehabilitation. This paper is concerned with the description and evaluation of our prototypic implementation of *Upbeat* that will serve as the basis for conducting clinical studies to evaluate its impact on rehabilitation.

## 1. Introduction

Limb loss is a recurrent problem all across the world. Every year, an estimated 185,000 people undergo upper limb amputations [1], and a significant portion of them add to the millions who live without the ability to comfortably perform activities of daily life (ADLs) [2, 3]. Efforts within the field have led to increased research in prosthetics over the years, enabling amputees to achieve higher degrees of motion and control aided with the development of myoelectric prosthetics. However, the functionality of these prosthetics remains limited, and coupled with the high rejection rate of these devices, development in the field has significant room for improvement.

A common cause of prosthetic rejection is unsuccessful rehabilitation therapy, in which the amputee is unable to develop the sufficient skills needed to successfully manage their prosthesis during ADLs [1]. Some of the major problems leading to rehabilitation failure include the late start of posttraumatic intervention due to wait time for a prosthetic fit, a lack of objective assessment of the patient's progress and performance [4], and poor patient motivation to commit to the repetitive practices involved in rehabilitation [5].

Augmented and virtual reality (AR/VR) has the potential to ameliorate the rehabilitation process. By using a virtual arm instead of waiting for a prosthetic, patients can start rehabilitation immediately after trauma, consequently reducing the acuteness of muscle atrophy [6]. An example is Anderson and Bischofʼs system, who developed an AR system involving a virtual arm overlaid on a patient's residual limb and controlled by residual limb muscle activity [7]. This system, when compared to traditional, non-AR game-based systems, showed higher user experience and investment as well as comparable muscle isolation. Furthermore, the advantage of the virtual arm enables the patient to start the rehabilitation process earlier.

Another issue with current rehabilitation in upper limb amputees is the lack of a comprehensive objective assessment of the patient's progress. Commonly used methods to evaluate patient progress include the Box and Block Test (BBT) [8], the Southampton Hand Assessment Procedure (SHAP) [9], and the Clothespin Relocation Test (CRT) [10]. However, these are standardized tests only evaluating performance within a small range of movement tasks with limited degrees of freedom (DOF). Their assessment methods only account for completion rate (number of tasks successfully accomplished), lacking a more comprehensive quantitative and qualitative assessment of the patient's performance. Monitoring run-time dynamics to provide a more comprehensive assessment is important for practitioners to evaluate how well the patients are restoring mobility [11].

Among the solutions to tackle the lack of comprehensive assessment mentioned above stands the protocol developed by Chadwell et al. [1], which combines EMG signal monitoring, kinematic sensing using inertial measurement units (IMUs), and gaze tracking to determine the patient's proficiency of using an upper limb prosthesis. The results provide information on the quality of movement as well as the completion rate and are highly regarded for both its incorporation of gaze tracking as well as for accounting for the unpredictability introduced by the skin-electrode interface. However, despite these novel features, this protocol had a duration of approximately 4 hours, which was inconveniently long for efficient clinical use [1].

A year later, Hunt et al. developed the Prosthetic Hand Assessment Measure (PHAM), an alternative method to quantitatively assess performance in a range of manipulation tasks associated with object manipulation (e.g., pinch, key, and power, shown in Table 1) for upper limb amputees [12]. PHAM uses IMUs for motion tracking and presents a performance evaluation assessment metric that accounts for compensatory movements in the patient. Another method proposed by Yu et al. utilizes a Kinect-based system to introduce a personalized range of motion measurement with AR feedback [13]. The goals of the study were to establish the accuracy of the Kinect in measuring clinically relevant movements in patients with Parkinson's disease. The results of this system match expertsʼ observations and show promising results for telerehabilitation scenarios [13], as well as, once again, the potential of rehabilitation within an AR system. As shown in the study by Yu et al., as well as later in *Upbeat*'s implementation, integration of motion tracking and electromyography (EMG) sensors within an AR system provides quantitative data physicians can use for objective assessment of patient progress. The flexibility of such a system also allows the therapy to be personalized to each patient's unique needs.

In addition to late posttraumatic intervention and lack of comprehensive assessment, one of the final main challenges of upper limb rehabilitation is maintaining patient motivation and commitment to practice, especially considering the prolonged and repetitive nature of this task. Previous work on gamified systems for AR-guided rehabilitation includes *mirrARbilitation* [14], a system based on gesture recognition and markerless motion tracking which recognizes and classifies biomechanical movements. The application provides exercise instructions, to prevent cheating via movement compensation, and has been proven capable of increasing patient success rate during rehabilitation, preventing wrong movements, and fostering an incentive to complete the process [14].

As such, AR/VR-guided rehabilitation proves to be effective in increasing motivation and adding excitement to rehabilitation practices, consequently leading to increased investment by the patients themselves. Similar results have been extensively studied in rehabilitation for stroke patients [6], results which remain highly applicable towards upper limb rehabilitation programs [15]. Altogether, the advantages of integrating AR into rehabilitation therapy lead to a more effective restoration of mobility in amputees by providing more accurate performance evaluation methods, providing real-time guidance for improved performance, and increasing patient's excitement and motivation while performing therapy.

*Upbeat* takes the rehabilitation workflow presented in PHAM [12] and incorporates it into an AR-based dance game, simulating the idea of practicing a set of different hand gestures within a dynamic environment. PHAM focuses on monitoring gesture completion rate and accounts for compensatory movement. In *Upbeat*, we expand upon this idea through monitoring of patient's EMG activity as well as providing an AR feedback visualization system that allows the patient to see the muscles activated throughout the gameplay. The proposed system shall be understood as a proof of concept in order to quantify performance and validate design decisions such that, upon completion of this study, a refined version of the system can be used to evaluate clinical appropriateness for rehabilitation on a control group of amputees.

## 2. Materials and Methods

The proposed system for rehabilitation is based on AR guidance, gesture recognition, and markerless body tracking. A virtual dance instructor guides the patient through a set of dance movements containing specific hand gestures (Figure 1). A Myo armband, worn on the forearm, is used to detect the patient's muscle activity and classify the hand gestures using detected EMG data. The patient's position is tracked with a Microsoft Kinect sensor and used to display a visualization of the muscle activity upon completion of the session. The system's workflow is described in Section 2.1 and summarized in Figure 2. Moreover, a detailed explanation of the materials and methods to develop each component in *Upbeat* is provided in Sections 2.2–2.6.

### 2.1. Game Workflow

The game is composed of three major scenes for each stage of the game—Menu (song selection), Play, and Feedback. Navigation throughout the application can be done with either mouse inputs or with gestures detected from the Myo Armband (Figure 3). The Play scene (Figure 1) is where the majority of the gameplay occurs. This scene has two key components: a dance instructor and a hand gesture prompt. The virtual dance instructor that appears on the side of the screen shows the patient the dance movements to follow. The virtual dance instructor is to give the patient visual cues on the correctness of their dancing and encourage continuous engagement, similar to a real-life dance instructor.

The hand gesture prompt is an image icon on the bottom right corner of the screen that informs the patient of which hand gesture to perform at the given moment. Hand gestures are tracked with the Myo Armband, and if the correct gesture is performed in the expected time frame, the image is replaced with a green success symbol to tell the patient that correct gesture is performed. In the final Feedback scene (Figure 4), the patient can see a visual summary of the data collected during gameplay. These data can also be sent to a rehabilitation practitioner for further analysis. The Feedback scene is displayed immediately after the Play scene, a few seconds after the completion of the song and choreography. An overview of the game's workflow is shown in Figure 2.

### 2.2. Game Development

*Upbeat* was developed with the 3D game engine Unity, through which all the sensors and software used (Kinect, Myo, *Mirracle* [4]) were integrated. The Myo Armband SDK for Unity was used to feed data from the Myo Armband sensor wirelessly into the Unity application. Additionally, the Kinect SDK for Unity was used to capture the pose and position of the patient during gameplay and to utilize the data into the postgame feedback. Along with a standard RGB video recorded during gameplay, motion data from the Kinect sensors were fed into *Mirracle* [4], an AR application used to produce a color-coded visualization of the patient's muscle activity during gameplay.

### 2.3. Dance Choreography

The integrated dance used in *Upbeat* was choreographed and recorded with the Kinect. The motion-capture data were then used to animate the in-game virtual dance instructor which later guides the patient through the same movements. The choreography consists of a set of dance movements embedded with hand gestures inspired by the PHAM model. The dance choreography was designed to include full range of motion in the upper body, as well as regular, repetitive movements. These two factors (movements with various degrees of freedom and repetitions) have proven to be beneficial in state-of-the-art rehabilitation therapies [12].

Each dance move includes one of the four hand gestures (spread, wave right, wave left, and fist; see Figure 3) and is performed in time with selected music—in this case, the current demo song is What About Us by P!nk. The song was chosen because it had a tempo appropriate for novice users to effectively engage with the game. Through repeated sessions, the patients learned the dance by following the virtual dance instructor while also practicing the hand gestures for rehabilitation.

In the PHAM protocol [12], the patient is required to manipulate a set of objects within a physical frame by grabbing the object and changing its position in the frame (see Table 1). Each object requires the patient to perform a particular hand gesture, as shown in Table 1. While the hand gestures included in the PHAM protocol are useful for object manipulation, in *Upbeat* we selected gestures common to activities of daily living (ADLs) (see Table 2). The gestures selected were spread, wave right, wave left, and fist (see Figure 3). These gestures were selected due to two key advantages: First, they are highly suitable for the EMG classification. Secondly, they can easily be embedded in dance choreography.

### 2.4. Motion Capture and Model Animation

The Kinect sensor, along with NI mate software, was used to capture the movements of a dancer performing the choreography. The NI mate software allowed the motion-capture data detected with the Kinect to be fed into Blender, a free open-source 3D creation suite (Foundation, Blender. “Blender.Org–Home Of The Blender Project–Free And Open 3D Creation Software,” Blender.Org, 2018, https://www.blender.org. Accessed 29 Nov 2018.), in the form of a rig, an animated 3D skeleton, which was later used to animate the dance instructor virtual model for the game (“Free Mannequin Male 3D Model.” Turbosquid.Com, 2018, https://www.turbosquid.com/3d-models/free-mannequin-male-3d-model/1005602. Accessed 29 Nov 2018.). The motion data from the NI mate rigging were matched to the model's body (Figures 5(a) and 5(b)). Because the visualization of specific hand gestures was for a correct practice, each of the hand gestures was manually key-framed in Blender (Figure 5(c)) to increase the accuracy and clarity of the model hand gesture visualization.

### 2.5. Gameplay Setup

The Myo Armband was placed on the upper arm of the patient, right below where the forearm is the widest. In the case of an upper limb amputee, this would correspond to the phantom limb. The Kinect sensor was positioned at an approximate distance of 1.5 meters in front of the patient and at a height aligned with their upper chest. A 43″ TV monitor was used to display the game and located at the same distance as the Kinect (1.5 m), which was a clearly visible location for the patient. In addition, speakers were connected to the computer and used to play the music for the dance game.

Before the gameplay begins, each user undergoes a calibration protocol for the Myo Armband to ensure correct hand gesture detection. Calibration is done through the Myo Armband's proprietary interface, *Myo Connect*. In the calibration, the user is prompted to perform each of the five recognizable gestures (wave in, wave out, fist, fingers spread, and double tap) a sequence of times. The process takes approximately 3-4 minutes overall, and it has to be done every time a new user interacts with the system.

The recording of the patient's performance during the game is displayed in real time on the game's background, simulating the effect of a mirror. This setup is the most appropriate in order for the patients to clearly see the virtual dance instructor, as well as their own mirrored reflection (from the head to slightly above their knees), such that they could perform the dance movements with as much visual observance as possible.

### 2.6. Performance Monitoring and Feedback

Performance consisted in three key elements: gesture completion, muscle activity, and muscle activation. The Myo Armband was integrated into the application to track EMG activity and detect the hand gestures. The gesture completion is evaluated using a score based on the number of successfully completed gestures. The patient's muscle activity is then shown using an EMG graph, while a color-coded visualization of muscle activation is produced with the *Mirracle* AR mirror system [4].

The postgame feedback is designed to deliver a comprehensive evaluation of the user's performance, following methods that have proven to be effective for rehabilitation [6, 12]. The purpose of the feedback is to serve the user with an immediate quantitative evaluation of how well they performed the gestures during gameplay (given by the Game Score), as well as a qualitative understanding of their movements through the color-coded visualization of their muscle's EMG data. This EMG graph also provides the practitioner with a detailed understanding of the user's current progress in regaining control of their upper limb muscles. The feedback components are shown in Figure 4 and explained further below.

#### 2.6.1. Game Score

The scoring system is based on the timing and accuracy of gesture completion. Each dance step shown by the virtual dance instructor contains one hand gesture that needs to be matched by the patient. Whether or not the patient successfully completes the gesture is tracked by the Myo Armband, which analyzes muscle activity in order to classify the movement into a recognized gesture. If the performed gesture both matches the one shown by the dance instructor and is performed within a certain time frame, it is deemed as the correct movement and adds 100 points to the player's total score. The time frame for each specific hand gesture and dance movement varies based on the choreography and music, but typically lasts between 6 and 12 seconds. The total game score is then calculated based on how many hand gestures are accurately performed by the player throughout the game, with points awarded for each successfully completed gesture.

#### 2.6.2. EMG Graph

The Myo Armband contains an array of 8 bipolar surface electrodes that measure the EMG activity from the user. The raw data are then streamed wirelessly through the Myo Data Capture application at a frequency of 200 Mhz to populate a.csv file (stored locally) that is later used to produce a graph of the patient's EMG activity.

This graph is displayed upon completion of the game in the Feedback scene. Each color in the graph represents data collected by each individual sensor, and the overall analysis can be used by the practitioner to visually analyze the muscle activity patterns as an indication of the patient's progress through the rehabilitation process.

#### 2.6.3. Color-Coded Visualization of Muscle Activity

In our system, the *Mirracle* application records a video of the patient performing the movements during the gameplay. It uses this video in combination with the Kinect depth sensor data to output the same video with an augmentation of the musculoskeletal system of the upper arm overlaid on top of the patient's right arm. The augmented muscles are color-coded (green for activated, red for relaxed) in real time to indicate the muscles being used.

## 3. Results and System Evaluation

The system was evaluated on three subjects, with 10 trials of the gameplay performed by each subject. In each trial, we measured the system's ability to correctly classify each specific gesture. Even though the classification is performed using the built-in Myo Armband software, measuring the classification accuracy within the *Upbeat* environment is important in order to evaluate whether or not the Myo Armband functions properly in a Unity environment.

For each trial, we also measured the system's operating time, reaction time, and detection time for each hand gesture involved in the gameplay. We define operating time (*o*_*t*_) as the time taken for each hand gesture to be detected by the system from the moment it appears on the screen. Operating time can be broken down into detection and reaction times (Figure 6, equation (1)). Detection time (*d*_*t*_) is defined as the time it takes for each specific gesture to be recognized by the system, while reaction time (*r*_*t*_) is defined as the time it takes the subject to perform a hand gesture from the moment it appears on the screen (Figure 6).

(1) $$\begin{array}{c} o_{t}=r_{t}+d_{t}. \end{array}$$

The results for each hand gesture class are shown in Table 3. Summarizing these results, the system reported an average detection time across hand gestures of 0.24 ± 0.31 seconds, while the average reaction time was 0.92 ± 0.10 seconds. Overall, this gives us an average operating time of 1.15 ± 0.34 seconds. We also calculated the classification accuracy, expressed as the percentage of correctly classified gestures per class across the 10 trials for each patient (Figure 7).

Since more advanced versions of *Upbeat* would involve faster dance movements expected to be performed within a shorter time period, it is crucial for the system to be able to detect different gestures quickly and accurately, in order to accommodate for the different levels of proficiency for each patient as their rehabilitation therapy progresses. To assess the system's ability to accommodate faster dance movements, we used the detection time data to compute the percentage of hand gestures that could be efficiently detected within a time interval of no more than four seconds (Figure 8). The results show that it takes an average of 2.62 seconds for each gesture to be detected, meaning the system could effectively support faster-paced choreography. To set this in context, Figure 9 shows the dance movement time interval across the current gameplay, which currently ranges between 6 and 12 seconds.

## 4. Discussion and Further Directions

From the experiments we conducted during our system evaluation, 77% of the gestures performed by the subjects during gameplay were detected and accurately classified by the system. Considering that the commercial Myo Armband has an average classification accuracy of 82.8% [16], *Upbeat's* results show that integrating the Myo Armband within *Upbeat's* local environment slightly compromises the classification accuracy.

Misclassification was more prevalent on the third subject. This was due to the difficulties this subject experienced during the calibration protocol, emphasizing the importance of a more robust calibration protocol compared to that of the commercial Myo Armband. Building a more robust calibration protocol and integrating it in the game's workflow with a tutorial/calibration feature are further steps for the system's improvement.

It is also important to consider that the hand gestures used in the current version of *Upbeat* have significantly differentiable EMG patterns. There is a trade-off between the complexity of the hand gestures and the accuracy of the EMG classification. If the sequence of hand gestures integrated in the game were to be expanded by introducing more complex hand gestures in a shorter time frame, the classification report of the system would be expected to achieve lower classification results. However, it is also expected that higher classification accuracy correlates with increased practice. The classification accuracy improves because, as the user becomes more experienced performing the rehabilitation exercises, the muscle signals become clearer and differentiable, which leads to better classification accuracy [12]. That is to say, as a patient becomes increasingly familiar with the choreography, it is expected that they can time and perform the gestures synchronously with the game with a higher degree of accuracy. As a result, this usage of gamified rhythm, time, and practice, likely contributes to higher success rates with the rehabilitative movements, making up for any initial complexity of the gestures. A further improvement to tackle this issue would be to add an initial learning session where the user learns the hand gestures and becomes familiar with the interface before the actual dance choreography begins.

Because the dance movements during gameplay take between 6 and 12 seconds (Figure 9), we expect that the system is able to detect the gestures faster than the minimum time of 6 seconds. With the purpose of assessing this, the reaction, detection, and operating times are measured and presented in Table 3 of the results section. Amongst the correctly classified gestures, the maximum detection time across trials was 2.62 seconds, which was well below the minimum of 6 seconds. However, we also had to take into account the reaction time, namely, the time between the appearance of the gesture symbol on the screen and the patient actually performing the gesture. In our study, the average reaction time was 0.92 seconds. By adding the detection time to the average reaction time, we can conclude that the operating time of the system is 3.56 seconds, which is still well below our minimum requirement of 6 seconds to perform a given movement. As such, we are certain that the current system is suitable for accurately recognizing gestures in a choreographed sequence. Given this operating time, there would still be room for the system to introduce more dynamic movements as part of more advanced levels.

*Upbeat* is a proof of concept aimed at testing whether a gamified, AR version of upper limb rehabilitation therapy, based on the PHAM protocol, could successfully be utilized in a clinical environment. Currently, we assert that the designed system and workflow is successful at classifying hand gestures embedded in a dance routine taught by a virtual dance instructor with a success rate of 77%. Furthermore, the system was also successful in measuring EMG signals from the patient's upper arm muscle activity, as reported by the graphical summary of the data as postgame feedback. Finally, the system was able to display a recording of the gameplay with an accurate augmentation of the musculoskeletal system overlaid over the patient's body, allowing the visualization of the muscles being activated during each dance movement.

In order to make the system appropriate for rehabilitation, the next step is to implement a more complicated set of hand gestures better reflecting those used in PHAM [12]. This process includes developing the Myo Armband built-in classifier to detect a broader set of hand gestures given the raw EMG data. Another improvement of the proposed system is adding different levels to the current version of *Upbeat*, where the difficulty is based on the speed of the music, the complexity of the choreography, and the range of movements involved. Additionally, analyzing the motion between poses and accounting for the compensatory movements in the scoring system would give a further insight into the patient's performance, for example, calculating the actual accuracy of the performed gesture (as opposed to the currently binary system of whether or not the gesture was completed).

Most importantly, a clinical study with a group of upper limb amputees shall be conducted in order to evaluate their progress when using *Upbeat* in comparison to that of a control group following traditional rehabilitation therapy. As the system is intended to improve rehabilitation in upper limb amputees, it is important to understand how a system like *Upbeat* is received by its target group. Furthermore, while the qualitative and analytical aspects of the system already have strong support, both from this study as well as related studies, a more subjective assessment on how enjoyable an application like *Upbeat* will be is a future target of study.

## 5. Conclusions

*Upbeat* converts the proven success of PHAM rehabilitation therapy and transforms it into a fun and enjoyable gamified experience for rehabilitation. As such, the gamified aspect of *Upbeat* has the potential to improve the rehabilitation process by increasing user's excitement. Portability of the system allows for rehabilitation to begin immediately after trauma, rather than waiting for prosthetics to be made or for medical-guided therapies to be concretely established. *Upbeat* further facilitates the important element of personalized feedback which can prove to be essential for the amputee to understand their progress, as well as giving doctors the ability to simultaneously track the progress without being overbearing on the rehabilitative process. *Upbeat* is presented as a prototype for gamified AR rehabilitation therapy and, in future work, will be used to conduct a clinical trial to evaluate its efficacy in achieving the envisioned goals.

## Figures and Tables

**Figure 1:** *Upbeat*'s gameplay screen.

**Figure 2:** Overview of *Upbeat*'s game navigation.

**Figure 3:** Hand gestures included in the choreography and tracked with Myo Armband (“Getting Starting With Myo On Windows”. Welcome To Myo Support, 2018, https://support.getmyo.com/hc/en-us/articles/202657596-Getting-starting-with-Myo-on-Windows. Accessed 29 Nov 2018.).

**Figure 4:** Feedback screen.

**Figure 5:** (a) NI Mate rig with motion-capture data using Kinect; (b) Blender model used for virtual dance instructor. (c) Manual keyframing of the model's hand bones with motion-capture data.

**Figure 6:** Detection time (*d*_*t*_) and reaction time (*r*_*t*_) measured during gameplay.

**Figure 7:** Hand gesture classification accuracy. This figure indicates the percentage of the gestures correctly classified across 10 trials, for each of the three users.

**Figure 8:** Optimal dance movement time interval. This figure reflects the percentage of hand gestures that would be detected, given different time interval thresholds in the range 0–4 seconds.

**Figure 9:** The time interval for each dance movement in the gameplay. Throughout the gameplay, there are sets of 10 movements, each containing one hand gesture.

**Table 1:** Correspondence of object, hand gesture, and ADL used in the PHAM method [12].

Object	Hand gesture	Activity of daily living (ADL)
Cylinder	Power	Pouring a glass of water
Prism	Tripod	Picking up a pencil
Block	Pinch	Picking up coins
Card	Key	Grasping a credit card

**Table 2:** Correspondence of hand gestures involved in *Upbeat* with ADL.

Hand gesture	Activity of daily living (ADL)
Spread	Greeting someone, offering help
Wave right	Indicating direction (right)
Wave left	Indicating direction (left)
Fist	Gripping a small object

**Table 3:** System's average, maximum and minimum detection, reaction, and operating times.

	Wave left	Wave right	Fist	Spread
Average detection time (s)	0.06 ± 0.09	0.06 ± 0.05	0.34 ± 0.52	0.49 ± 0.68
Maximum detection time (s)	0.38	0.17	2.20	2.62
Minimum detection time (s)	0.02	0.02	0.02	0.02
Average reaction time (s)	0.88 ± 0.28	1.09 ± 0.47	0.87 ± 0.49	0.83 ± 0.36
Maximum reaction time (s)	1.53	2.02	2.55	1.33
Minimum reaction time (s)	0.22	0.05	0.02	0.03
Average operating time (s)	0.94 ± 0.37	1.14 ± 0.53	1.20 ± 1.00	1.33 ± 1.04
Maximum operating time (s)	1.92	2.18	4.75	3.95
Minimum operating time (s)	0.23	0.07	0.03	0.05

## Data Availability

Release of source code and data will be considered on a per request basis.

## Supplementary Materials

Supplementary Materials Supplementary Material shows a demo video of the system. The user first selects the “start” option in the menu and browses through the available songs for the gameplay. This control is enabled by the Myo Armband, worn on the forearm, which detects the patient's muscle activity. Once the song has been selected, the gameplay starts and the virtual dance instructor (shown on the left of the screen) shows the user the dance movements to imitate. The hand gesture prompt is an image icon on the bottom right corner of the screen that informs the patient of which hand gesture to perform at the given moment and whether this is performed correctly. The labels on the top of the screen display the current score on the left and time left for the gameplay on the right. Finally, an additional view of the user during *Upbeat* gameplay has been added in the top right corner to give a better understanding on the system's setup and the placing of the webcam.
